This article has been retracted.

# Forecasting the transportation energy demand with the help of optimization artificial neural network using an improved red fox optimizer (IRFO)

**DOI:** 10.1016/j.heliyon.2023.e21599

**Published:** 2023-11-02

**Authors:** Yijie Liu, Gongxing Yan, Andrea Settanni

**Affiliations:** a Chongqing Creation Vocational College, Yongchuan 402160, Chongqing, China; b School of Intelligent Construction, Luzhou Vocational and Technical College, Luzhou 646000, China; c Luzhou Key Laboratory of Intelligent Construction and Low-carbon Technology, Luzhou 646000, China; d University of Tirana, Tirana, Albania; e College of Technical Engineering, The Islamic University, Najaf, Iraq

**Keywords:** Optimization, Energy demand, Transportation, Optimize ANN, GDP

## Abstract

Transportation energy demand has a significant impact on worldwide energy consumption and greenhouse gas emissions. Accurate transportation energy demand predictions can help policymakers develop and implement successful energy policies and strategies. In this study, a novel approach to predict transportation energy demand using the Artificial Neural Network (ANN) based on the Improved Red Fox Optimizer (IRFO) has been suggested. The proposed method utilizes the ANN model to solve the complex nonlinear relationships between transportation energy demand and its effective parameters including Gross Domestic Product (GDP), population, and vehicle numbers. Also, the IRFO algorithm was utilized to modify the ANN model's parameters to improve the prediction accuracy. The experimental findings demonstrate the ANN-IRFO model performs better than the other method in terms of accuracy and effectiveness. It predicts the growth of GDP, population, and vehicles number by 5.5 %, 4.8 %, and 4.2 %, respectively. The findings demonstrate that the suggested method can provide accurate forecasts for transportation energy demand, which can help decision-makers to make informed decisions and policies regarding energy management and sustainability.

## 1 Introduction

Transportation is one of the most important economic sectors [1]. Today, transportation is one of the most important fields of service in any country, so its development is a sign of progress in any country [2]. This means that any country with a better-equipped and more efficient transportation system is more economically advanced [3]. Thus, there is a two-way relationship between economic development and the expansion of transportation services [4]. According to the available statistics and information, the transportation sector is one of the largest consumer sectors [5]. The transportation sector is also the main consumer of petroleum products, which is growing with the development of countries [6]. Among the transports, land transportation (road and rail) is the most important branch of transportation [7]. This sector has the highest share in terms of passenger and goods movement and the highest consumption of energy in the transport section [8].

The important issue in the transportation sector is energy demand [9]. Petroleum is used to satisfy most of the energy needs in the transport section [10]. Therefore, one of the important features of the transportation sector is fuel consumption, which is one of the main intermediate goods in the production process [11]. Following economic growth in populous countries, the range of energy demand will increase, so fuel consumption for transportation will increase significantly due to increased demand [12]. These days, energy provision has been one of the most basic requirements for the country's breakthrough from a social and economic perspective. Alterations in urbanization and demographics, as well as weaknesses in transmission efficacy and distribution, increase energy demand, rapid consumption of resources, and lack of dependence on clean energy sources [13].

The growth and survival of economic activities in countries depend on energy. Therefore, the governments of the countries try to have accurate planning in the direction of energy consumption and demand through more accurate predictions [14]. Also, they can control the parameters of energy supply and demand optimally [15]. Analyzing the factors affecting the intensity of energy consumption, demand growth, and prediction of them, allows managers to take the necessary actions to control energy supply and demand variables [16].

It is necessary to study the parameters affecting energy demand in the process of transportation services through different methods [17]. Intelligent systems, especially Neural Networks (NNs) due to their successful performance in the field of diagnosis and model identification are used in many prediction problems [18]. Nowadays, utilizing intelligent technologies to find a solution for complicated practical issues in the departments of different activities has captured attention on an unprecedented scale. Learning general rules is available for these systems with the aid of some computation based on empirical information [19].

Artificial Neural Networks (ANNs) have been categorized as intelligent systems with understanding embedded in them. The empirical data has been transferred to the structure of the network by them [20]. The prevalent benefit of ANNs is their capability to model complicated relationships that are not linear, regardless of previous assumptions [21]. It is very important to predict the trend of energy demand to adopt appropriate policies. Because of the volatile, nonlinear inclination of energy need and the factors influencing it, intelligent and nonlinear capabilities, especially ANNs, to predict energy demand have been proven in proven studies.

Much research has been done on forecasting energy demand that could be referred to by Di Leo et al. [22] demonstrated the use of regression analysis to forecast energy demand patterns in end-use industries. The suggested approach is used to define the links between population and GDP (independent variables) and residential, transportation, and commercial energy needs. Classical statistical tests have proven the usefulness of linear and nonlinear regression frameworks for electricity demand prediction. Energy demand estimates were validated as input data to the bottom-up TIMES algorithm in the two scenarios, proving the projection technique's validity. The limitation of this study was the use of two variables, population, and GDP, to predict energy demand, because these variables as independent factors cannot consider all the variables affecting energy demand patterns. Therefore, inaccurate or insufficient information sources can lead to incorrect predictions. Also, the non-linear regression technique can predict energy demand depending on the studied areas and is limited to the studied time horizon.

Hao et al. [21] used a new method for predicting energy demand called the Artificial Bee Colony (ABC) Algorithm. This research proposed and implemented a unique ensemble prediction model for energy consumption based on the Artificial Bee Colony (ABC) algorithm. This model was developed and evaluated using China's primary energy demand data. The findings showed that the proposed approach of benchmark forecasting techniques and simple average forecasting method performs better in terms of accurate forecasting and hypothesis testing, and the ensemble algorithm forecasts for the coming years show that China's future electricity demand will maintain a steady growth trend. The successful implementation of the suggested model, which cannot be transferred to other nations or areas, is a limitation of this research. It is assumed in this study that the connection between energy demand and the input parameters is linear and that the ABC algorithm can detect essential patterns and trends. The accuracy of the predictions, however, might be restricted by the quality of the data utilized, and it is difficult to comprehend and define due to the complicated structure and application of the ABC algorithm.

Fani et al. [23] applied the multilayer perceptron neural network to social and economic indicators to model energy demand forecasts in the transport sector. In this study, the scenarios were presented based on a pessimistic and optimistic view of energy demand by 2020. The following factors are used to forecast power demand: The Gini coefficient, fuel price, average household income, population, hybrid/gasoline car ratio, average vehicle, the price index of products and services, and lifespan. The average percent error was found to be 3.8 % and 4.6 %, respectively. The ratio of hybrid and gasoline automobiles, population, and average vehicle lifespan all had a significant effect on gasoline usage, according to sensitivity analysis. The result of the energy demand forecast based on three scenarios for four years was provided. The results of the forecast showed that if the current trend of economic and social variables continues, energy demand in the transport sector will increase. The present study has a limited number of factors to forecast energy demand, which can be limited by the quality of the sources of data. Additionally, the efficiency of the model can be restricted to the specific time interval and geographic region investigated, and its forecasts may be susceptible to uncertainty due to unforeseen incidents or changes in external elements.

Nabavi et al. [24] used machine learning models for household and commercial electricity consumption. This research predicts commercial and household electricity consumption in Iran using three machine learning techniques: multiple linear regression, multiple logarithmic linear regression, and nonlinear auto-regression with artificial neural networks with exogenous input. To predict energy consumption, factors such as GDP, population, natural gas prices, and electricity prices were used. The results showed that Iran's household and commercial energy consumption will be 76.97 %, 96.42 %, and 128.09 Mtoe, respectively, until 2040. These findings show that Iran should design and implement new policies to increase the percentage of renewable energy sources in total energy consumption. In this study, the use of a limited number of energy demand forecasting variables may not be enough to cover all relevant factors. The precision of energy demand approximations and input data may be limited by the caliber of the data sources. Machine learning techniques may be limited to a specific geographic area and time frame, and projections may be indeterminate due to unforeseeable occurrences.

Del Real et al. [25] investigated the use of deep learning algorithms to predict electricity consumption. This study presented a hybrid design that included a Convolutional Neural Network (CNN) with an ANN model. Using ARPEGE forecast meteorological data, the proposed framework was trained and applied in an actual situation to produce a forecast of French electricity consumption. Compared with other methods such as Automatic Moving Mean Regression (ARIMA) and classic ANN, the findings showed that this strategy beat the reference RTE subscription-based service and achieved the highest performance score. The performance of the model was assessed using only one real situation and may not be important to other conditions or areas. Information value, assumptions, generalizability, ambiguity, and a lack of explanation are all problems that might stymie its practical use and uptake. The research's hybrid design may not apply to other areas or historical periods.

Zeng et al. [26] attempted to predict energy consumption using an integrated intelligent technique called ADE-BPNN, a Back-Propagation Neural Network (BPNN) model backed by an adaptive differential evolution algorithm. As inputs, the suggested combined model integrates GDP, population, import, and export statistics. To improve the BPNN's forecasting performance, enhanced differential evolution with adaptive mutation and crossover is used to identify acceptable global starting connection weights and thresholds. The findings showed that the proposed ADE-BPNN performs better than other models. This model predicts energy consumption with the most accurate due to advanced adaptive DE with a good balance of search speed and accuracy. The use of the ADE-BPNN model in this work results in a limited range of variables, poor data quality, assumptions, generalizability, uncertainty, and minimal explanation. The model assumes a certain amount of linearity or nonlinearity between the input and output variables; nevertheless, it should be emphasized that the real connection between these variables is not always clearly evident. It is critical to recognize that the model's forecasts may be compromised owing to unanticipated occurrences or alterations to external elements that were not considered during its formulation.

Peng et al. [27] utilized effective energy consumption forecasting using empirical wavelet transforms and long short-term memory. Energy consumption is an important issue of global concern. Accurate energy consumption forecasting can help balance energy demand and production. Although there are various energy consumption forecasting methods, their accuracy still needs to be improved. This study applied a long short-term memory-based model to energy consumption forecasting to achieve better prediction performance, and the more critical influencing factors are emphasized. Results of one comparative example and two extended applications show the proposed model achieves better prediction accuracy compared with basic long short-term memory and other existing popular models. The mean absolute percentage errors of the proposed model for three real-life cases are 4.01 %, 5.37 %, and 1.60 %, respectively. Therefore, the proposed model is a satisfactory method for energy consumption forecasting due to its high accuracy. High-precision forecasting technology is important for the energy system. The ability of the framework was examined using just one comparison example and two expanded applications, and its usefulness may be restricted to the specific data utilized for its construction and assessment. The model's complexity, data quality, assumptions, generalizability, uncertainty, and inadequate explanation make it challenging to evaluate and explain. It might not apply to different circumstances or areas.

The primary objective of this paper is to forecast energy demand in the transportation industry. In comparison to previous research, this study proposes an improved technique for estimating energy demand in the transportation industry. This technique is developed from Artificial Neural Network (ANN) based on the Improved Red Fox Optimizer (IRFO). Although the research literature shows that the use of optimization approaches in artificial neural networks may increase the accuracy of energy demand forecasting, it should be considered that optimization techniques can also cause prediction problems due to some optimization shortcomings. One of the optimization technique's shortcomings is that they tend to get trapped in the local optimal region, resulting in early convergence of the optimization technique, which may hinder finding a solution to the problem. The proposed technique tackles the drawbacks of optimization methods by providing the LF method (Lévy flight) and a circular mapping-based chaos mechanism. Therefore, improving the accuracy of energy demand simulation in the transportation sector allows managers to plan satisfactorily to supply electricity resources and meet society's demand.

Therefore, the main contribution of this study can be briefly highlighted as follows.

• The transportation energy demand forecasts by an optimized ANN model
• The Improved Red Fox Optimizer (IRFO) was used to optimize the ANN model.
• The GDP, population, and vehicle numbers are used to forecast.
• The ANN-IRFO model optimizes parameters to improve forecasting accuracy.
• The ANN-IRFO model provides reliable forecasts for transportation energy demand.

## 2 Method and material

### 2.1 Artificial neural network (ANN) model

An ANN is a simplified model of a central mechanism modeled on the brain structure. This method uses complex computational structures within neural neurons to give them the ability to respond to changes and adapt to the data environment. A Neural Network (NN) is an interconnected set of neurons set in diverse layers that are in touch with others by sending information [28]. There have been 3 layers in the mentioned model: input, middle, and outer, each of which has its specific tasks. Input neuron information is used to generate output neuron information. The middle neurons are also responsible for processing this information. In general, the artificial neural network acts as a function and receives the input variables in several input layers. After processing and calculating the desirable goal, the output variables and the number of output layers are presented. In the mentioned approach, the neurons of the input layer receive socioeconomic variables values. The neurons of the middle layer forecast the values of transportation energy demand utilizing the procedures of trial-and-error (T&ER). Lastly, the neurons of the outer layer give the outcomes of the transportation energy demand prediction [29]. The correlation between the middle and input layers and the output by weight indicates the relative importance of the layers in calculating the output value. Each neuron has a certain weight. There are two types of weights in the ANN model: *a*_*j, i*_ hows the input layer weight, and *a*_*k j*_ define the output layer weight.

The transportation energy demand forecasting is evaluated in 2 steps. The 1st step calculates the sum of the weights of all input data (equation (1)):

(1) $$X_{i}=\sum_{j=1}^{m}a_{ij}N_{i}+B_{i}$$

where, $N_{i}$ shows several input data, $B_{j}$ does describe the middle layer weight bias, $a_{ij}$ shows the weight of the input layer.

In the 2_nd_ step, the determination of the output layer is implemented. Different types of activation functions are used to give the output results. In this study, the sigmoid function has been utilized and calculated using equation (2):

(2) $$F_{j}\left(x\right)=\frac{1}{1+e^{{-F}_{j}}}$$

Finally, the output calculates with the help of equation (3):

(3) $$Y_{i}=\sum_{j=1}^{m}a_{kj}N_{j}+B_{j}$$

Fig. (1) shows the structure of an ANN model.

**Fig. 1:** The structure of an ANN model.

Nevertheless, the artificial neural network is a powerful soft computing tool for forecasting transportation energy needs and is capable of being improved with the aid of optimizing algorithms. Presenting an appropriate action plan to achieve optimal system performance in any situation is defined as optimization [30]. More accurate results can be obtained in predicting transportation energy needs through the optimal selection of the input variables (initial weight), the intermediate layers’ quantity, and a proper optimization technique. The use of optimization processes is necessary to obtain satisfactory results. Transportation energy demand forecasting is a complex process. Therefore, classical methods can increase the prediction error. Recently, the mathematical basis algorithms used to optimize the ANN model, and the metaheuristics algorithms have been utilized regularly for solving the complication of optimization issues. In this research, a novel metaheuristic optimizing algorithm is suggested to optimize the ANN model. To simulate the software MATLAB 2016 is employed for optimizing the artificial neural network model in this paper. This procedure is explained in the following sections.

### 2.2 Optimization technique

#### 2.2.1 The optimization conception

The purpose of optimizing the process is to discover a proper solution to the problem, which could be a qualitative or quantitative conception [31]. Optimization is a technique for resolving a mathematical fitness function to determine the ideal quantity in engineering problems [32]. This optimal value can be minimum or maximum depending on the goal [33]. To determine the optimal amount, several studies have been performed [11]. For instance, traditional approaches included gradient lowering operations and the Pontryagin methodology provided the best and most accurate solution to such problems [31,34,35]. However, due to some optimizing issues' complexity and the incapability of classical ways to resolve these complicated problems, classical methods are less frequently applied [36]. Recently, researchers have developed novel techniques for solving optimization issues called metaheuristic approaches [35,37]. Metaheuristic algorithms can solve complex optimization problems based on random solutions [38], and are one of the most successful methods for predicting energy demand [39]. They are triggered by wildlife, sports, animal manners, and humans [40]. Metaheuristics are constantly evolving and improving [41]. Such as Genetic Algorithm (GA) [22], Spotted Hyena Optimizer (SHO), Multi-verse Optimizer (MVO) [42], and the original Red Fox Optimize (RFO) [17].

In this study, a newly found nature-inspired algorithm known as Red Fox Optimize (RFO) will be applied to improve energy demand forecasting. The RFO is a nature-inspired optimization technique used to solve complex optimization problems. Although other intelligent algorithms are available, RFO is often chosen due to its unique method of optimization and its ability to deal with a wide variety of challenges. RFO is an intelligent method that can manage both continuous and discrete parameters. Also, Also, the implementation of this algorithm is somewhat easier because it is not necessary to have programming experience or a comprehensive grasp of complicated mathematical ideas. These advantages make the algorithm accessible to a variety of users, including those who may not have a background in machine learning or optimization.

#### 2.2.2 The Red Fox Optimizer (RFO)

These types of foxes have been the pamphlets of carnivores. Their shape is narrow and elongated, which is due to their ease of running and chasing targets. The ears of this creature are sharp, and its head is long. Foxes are small—about 80 cm. They have relatively short legs and hairy tails. This animal has two standards of living. Some live in a certain habitat; however, some live nomadically and are constantly changing their place of residence. In both lifestyles, group leadership is headed by alpha couples. In these groups, each fox is capable of leaving the set after growing up and forming its territory or inheriting the territory of its parents. The key nutrition source for the foxes is tiny animals and pets. These creatures approach the prey by hiding and try to trap the prey by crawling toward it.

Fig. (2) presents the modeling of the fox shooting process in the optimizing procedure.

**Fig. 2:** The hunting process of fox in the optimizing approach.

The technique has two principal components: zone exploration, and the fox victim selection model. In cases of exploitation, the fox approaches the prey as far as it is possible to catch it. To initialize the algorithm, we must first present a few individuals from the swarm that is produced on a random basis. Assuming x is the primary swarm, we must (equation (4)):

(4) $$\bar{x}=\left[x_{0},x_{1},\ldots ,x_{n-1}\right]$$

To define each fox $x_{i}$ in iteration t, it has been described as ${\left({\bar{x}}_{j}^{i}\right)}^{t}$, where i shows the number of population and j situations the issue dimension over the solution area. That is assumed, the individuals (foxes) make movements throughout the search space based on the formulas. Assuming $f\in R^{n}$ as the function of condition for n parameter, the bellow marks indicate points over the boundary of ${\left[a,b\right]}^{n}$ (equation (5)),

(5) $${\left(\bar{x}\right)}^{i}={[\left(x_{0}\right)}^{i},{\left(x_{1}\right)}^{i},\ldots ,{\left(x_{n-1}\right)}^{i}]$$

Here a,b∈R.

Therefore, ${\left(x\right)}^{i}$ is to be by far the most suitable solution, whenever $f\;\left({\left(x\right)}^{i}\right)$ provides the global optimal.

To search global optimal in the algorithm, the below procedures should be assumed. In a red fox's herd, all individuals perform their duties of helping the members in the wild. Individuals move to faraway parts for finding prey providing that the habitat no longer has sufficient prey. This is normally modeled on the objective amount of individuals. Accordingly, the swarm is sorted by their objective function amount, and for ${\left({\bar{x}}_{best}\right)}^{t}$. To perform this, the Euclidean distance square is obtained for the individuals according to the (equation (6)):

(6) $$D\left({\left({\left(\bar{x}\right)}^{i}\right)}^{t},{\left({\bar{x}}_{best}\right)}^{t}\right)=\sqrt{\left\|{\left({\left(\bar{x}\right)}^{i}\right)}^{t}-{\left({\bar{x}}_{best}\right)}^{t}\right\|}$$

Afterward, the candidates go through the most suitable result through the below formula (equation (7)):

(7) $${\left({\left(\bar{x}\right)}^{i}\right)}^{t}={\left({\left(\bar{x}\right)}^{i}\right)}^{t}+\alpha \times sgn\left({\left({\bar{x}}_{best}\right)}^{t}-{\left({\left(\bar{x}\right)}^{i}\right)}^{t}\right)$$

where α shows a random value.

Here, if the new situation has a more desirable answer compared to the prior situation, that is to be chosen as the renewed solution, otherwise, all agents are likely to return to the former situation. In this state, if the hunt's exact status is discovered, the explorers give the location information to the group, otherwise, they return “empty-handed”. It must be regarded that due to unfamiliarity with long-distance foxes, their capacity of hiding and escape has been smaller compared to their colony. It has been displayed by removing the worst-case procedure in any epoch. The foxes pass through their areas in prey search. If the fox sees its prey, it starts in the closest possible position in silence to avoid being seen. Finally, it hoops the prey and tricks it to show that he has no interest in the hunting process. Whenever it gets close to the prey, it moves fast as probable to take the victim. The method has been regarded as a section of the RFO exploitation.

μ is a random amount varied from zero to one, that is used to model the probability of a fox being sawed whereas moving closer toward the target, like (equation (8)):

(8) $$\left\{ \begin{array}{c} move\;closerif\mu >3/4\\ stay\;and\;hidei\mu \leq 3/4 \end{array}\right.$$

If throughout the epoch, μ shows a moving to the swarm an improved Cochleoid formula has been applied to visualize the candidates' movement.

To consider motion, the observation radius of the fox is assumed through 2 variables. a is the primary factor that defines an ascending parameter introduced for any agent for random simulating the varying interval for nearing the target. The parameter is a number that randomly changes in the range [0–2]. The next parameter is $\varphi_{0}$ that has been used for the agents whenever the procedure begins and does model viewing angle of the fox. This variable has been defined over the range of 0 and 2***π***. These variables have been applied and the fox observation radius has been obtained using the equation as (equation (9)):

(9) $$r=\left\{ \begin{array}{c} \frac{a\times \sin\left(\varphi_{0}\right)}{\varphi_{0}}if\varphi_{0}\neq 0\\ \gamma if\;\varphi_{0}=0 \end{array}\right.$$

where γ displays a random value that is between 0 and 1. This is defined as the contrary impact of weather circumstances such as fog and rain. The agents' motion has been modeled using the bellow formulas (equation (10)):

(10) $$\left\{ \begin{array}{c} x_{0}^{New}=a\times r\times \cos\left(\varphi_{1}\right)+x_{0}^{actual}\\ x_{1}^{New}=a\times r\times \sin\left(\varphi_{1}\right)+a\times r\times {\cos\left(\varphi_{2}\right)+x}_{1}^{actual}\\ x_{1}^{New}=a\times r\times \sin\left(\varphi_{1}\right)+a\times r\times \sin\left(\varphi_{2}\right)+a\times r\times {\cos\left(\varphi_{3}\right)+x}_{2}^{actual}\\ \vdots \\ x_{n-1}^{New}=a\times r\times \sum_{k=1}^{n-2}\sin\left(\varphi_{1}\right)+a\times r\times {\cos\left(\varphi_{n-1}\right)+x}_{n-2}^{actual}\\ x_{n-1}^{New}=a\times r\times \sin\left(\varphi_{1}\right)+a\times r\times \sin\left(\varphi_{2}\right)+\ldots +a\times r\times \sin\left(\varphi_{n-1}\right)+a\times r\times {\sin\left(\varphi_{n-1}\right)+x}_{n-a}^{actual} \end{array}\right.$$

Where, for the points, the angular have been randomized based on $\left[\varphi_{1},\varphi_{2},\ldots \varphi_{n-1}\right]$.

This behavior of the fox is modeled after nearing the prey to hunt when it goes quietly towards the prey, and it's repeated to try to obtain another victim under the circumstances that the 1st attack fails. In nature, the foxes have to cope with different threats. Because food might not be immediately available in its habitat, therefore, relocation is essential to find prey. One of these threats is humans. Because One of the prey of the red fox is a pet. Therefore, there is a possibility of tracking foxes by humans. In nature, however, not all foxes die and migrate. Most of them are very intelligent and can escape and reproduce, bringing new ways to fox herds. To model this practice, we selected five percent of the individuals that are the worst in the community on the basis of the benchmark function's amount. This amount has been applied as our personal opinion to simulate small changes in the herd per iteration. We assume that each of these red foxes has been transferred to another or caught by a hunter because they are the least fit. A habitat model is applied to be created by alpha pairs for replacing them with new agents to preserve the size of the population continually. The most desirable agents are chosen ${\left(\bar{x}\left(1\right)\right)}^{t}$ , ${\left(\bar{x}\left(2\right)\right)}^{t}$ to represent the alpha pairs in the RFO $t^{th}$ iteration, where, the center of the territory is calculated using the (equation (11)):

(11) $${\left(Hab^{center}\right)}^{t}=\frac{{\left(\bar{x}\left(1\right)\right)}^{t}-{\left(\bar{x}\left(2\right)\right)}^{t}}{2}$$

The distance of habitat on the basis of Euclidean distance is calculated as (equation (12)):

(12) $${\left(Hab^{diameter}\right)}^{t}=\sqrt{\left\|{\left(\bar{x}\left(1\right)\right)}^{t}-{\left(\bar{x}\left(2\right)\right)}^{t}\right\|}$$

We choose a random value, κ is between 0 and 1 through the iteration, that represents agents in the iteration and is calculated using the (equation (13)):

(13) $$\left\{ \begin{array}{c} New\;nomadic\;candidateif\kappa >0.45\\ Reproduction\;of\;the\;alpha\;coupleif\;\kappa \leq 0.45 \end{array}\right.$$

Initially, it is assumed that the new members of the group leave their living place as nomadic animals to find nutrition and reproduce. In searching region, out of the living place, situations are randomly opted. Afterward, the new agents have been made using the alpha couple, therefore, we generate two of the more suitable members ${\left(\bar{x}\left(1\right)\right)}^{t}$, ${\left(\bar{x}\left(2\right)\right)}^{t}$ as a renewed individual (${\left({\bar{x}}^{rep}\right)}^{t}$) (equation (14)).

(14) $${\left({\bar{x}}^{rep}\right)}^{t}=\kappa \frac{{\left(\bar{x}\left(1\right)\right)}^{t}-{\left(\bar{x}\left(2\right)\right)}^{t}}{2}$$

#### 2.2.3 Improved red fox optimizer (IRFO)

The Red Fox Optimizer *(*RFO) is one of the latest techniques for optimization. Nevertheless, there are numerous advantages of this method that can be applied to resolve diverse types of optimization issues. In some problems, it could lead to early convergent results. Such an occurrence could be seen in optimizing several benchmarks in the defaulting article [43]. Lately, numerous techniques have been presented using chaotic maps for developing the techniques of optimizing efficiency. As mentioned, κ in the RFO is a random parameter, whereby utilizing iteration, the optimizer is more likely to converge early.

In the represented study, a circular mapping-based chaos method is applied to solve this problem. This method describes the variable κ as a regular formula with the help of the (equation (15)) [44]:

(15) $$\kappa_{i+1}=\kappa_{i}+\beta -\left(\alpha -2\pi \right)\sin\left(2\pi \kappa_{i}\right)\mathrm{mod}\left(1\right)$$

Here, a disordered time sequences $\kappa_{i}\in \left[0,1\right]$ have been made using considering $\alpha =\frac{1}{2}$ and $\beta =\frac{2}{10}$.

The research has applied the LF method (Lévy flight) for increasing finer convergency. This method shows a common method in the optimization method [45]. This function does simulate the random march for governing the local search using the (equation (16), (17), (18)) formula:

(16) $$\text{Le}\left(w\right)\approx \frac{1}{w^{1+\tau }}$$

(17) $$w=\frac{A}{{\left|B\right|}^{1/\tau }}$$

(18) $$\sigma^{2}={\left\{\frac{\Gamma \left(1+\tau \right)}{\tau \Gamma \left(\left(1+\tau \right)/2\right)}\frac{\sin\left(\pi \tau /2\right)}{2^{\left(1+\tau \right)/2}}\right\}}^{\frac{2}{\tau }}$$

Here, Γ(.) shows the function titled Gamma, τ defines the LF index varied from zero to two (here, $\tau \text{is}\;\text{equal}\;\text{to}\;\frac{3}{2}$ [46]), $A/B∼N\left(0,\sigma^{2}\right)$ shows the made samples using a Gaussian distribution, whereby mean is 0 and $\sigma^{2}$ is variance, respectively.

Using the method of LF, the renewed situations of the agents have been calculated based on the (equation (19)):

(19) $${\left({\left(\bar{x}\right)}^{i}\right)}_{New}^{t}={\left({\left(\bar{x}\right)}^{i}\right)}^{t}+\alpha \times sgn\left({\left({\bar{x}}_{best}\right)}^{t}-{\left({\left(\bar{x}\right)}^{i}\right)}^{t}\right)\times \text{Le}\left(\delta \right)$$

#### 2.2.4 Verification of algorithm

The efficacy of the improved RFO will be confirmed in comparison with other algorithms in this part. To represent a certain comparison, five different test function is used. Table 1 illustrates the employed test functions as well as their acceptable mount ($f_{\min}$) and their limitation for the evaluation [47].

**Table 1:** Test functions and their acceptable amount ($f_{\min}$) and their limitation for the evaluation [47].

Function	Range	$f_{\min}$
$F_{1}\left(x\right)=\sum_{i=1}^{n}x_{i}^{2}$	[-100,100]	0
$F_{2}\left(X\right)=\sum_{i=1}^{n-1}\left[{\left(x_{i}+0.5\right)}^{2}\right]$	${\left[-100,100\right]}^{n}$	0
$F_{3}\left(x\right)=\sum_{i=1}^{n-1}\left[100{\left(x_{i+1}-x_{i}^{2}\right)}^{2}+{\left(x_{i}-1\right)}^{2}\right]$	[-30,30]	0
$F_{4}\left(x\right)=\sum_{i=1}^{n}{ix}_{i}^{4}+random[0,1)$	[-128,128]	0
$F_{5}\left(X\right)={\left(x_{2}-\frac{5.1}{4\pi^{2}}x_{1}^{2}+\frac{5}{n}x_{1}-6\right)}^{2}+10\left(1-\frac{1}{8\pi }\right)\cos\;x_{1}+10$	${\left[-5,15\right]}^{2}$	3979

Also, the outcomes are compared with the help of numerous optimization approaches, such as Genetic Algorithm (GA) [48], Multi-verse optimizer (MVO) [49], Spotted Hyena Optimizer (SHO) [42], and the original Red Fox Optimizer (RFO) [43]. For the investigated methods, the set parameters have been illustrated in Table 2 [50].

**Table 2:** The setting variables for the studied optimizers in this research [50].

Approach	Parameter	Amount	Approach	Parameter	Amount
MVO [49]	Distance ratio of traveling	[0.6, 1]	GA [48]	Generations' quantity	100
	Existence possibility of a Wormhole	[0.2, 1]		Size of Population	100
				Type of Crossover	One cutting-point crossover
SHO [42]	$\vec{M}$	[0.5, 1]		Possibility of Crossover	$\frac{8}{10}$
	$\vec{h}$	[0,5]		Type of Mutation	Strong

Simulation is implemented in the MATLAB R2016B software environment. The simulation is implemented 45 times freely for any optimization approach and test functions to represent trustworthy outcomes for comparisons. To represent a reasonable assessment, for all methods, the size of the population is selected 100 with 400 repetitions for the entire studied algorithm.

### 2.3 The ANN/IRFO model development and application in transportation estimation demand

#### 2.3.1 The ANN/IRFO model development

One of the general methods to reduce the error value in the training of artificial neural networks is to use the Back Propagation (BP) process. As mentioned in the previous description, the BP method is utilized to train of artificial neuron network. The BP method is used to reduce the gradient. One of the main shortcomings of the BP technique is that it is prone to being easily stuck into the local minimal to reduce the gradient. These shortcomings cause several complicated issues in the results’ pattern identification. For solving this difficulty, numerous techniques have been suggested. In this research, to resolve this problem instead of reducing the gradient, a new method of combining ANNs and an improved optimizer has been represented. The ANN/IRFO model includes two main parts.

1) Artificial Neural Networks (ANNs).
2) IRFO algorithm that has been designed as a model to achieve ANN weight optimization.

There are two main purposes for applying IRFO in the ANN method.

1) Choosing proper fitness performance
2) Select the search factors.

Therefore, IRFO-based ANN as.

1) Compute the initial Red fox quantity in weight a and assess the cost function.
2) Renew the present act status for cost function amount on the basis of the Red fox prey and distance from the prey.
3) Verify that the network has obtained a satisfactory error value.
4) If the criteria condition is not identified, go to the stage (2).
5) If you have the necessary conditions:
6) End

MSE (Mean square deviation) is utilized to evaluate the ANN error. The main objective of MSE utilization is to estimate the disparity between acceptable and actual amounts. The MSE is calculated based on the (equation (20)):

(20) $$MSE=\frac{1}{m}\;{\sum_{i=1}^{n}\sum_{j=1}^{m}\left(x_{j}\left(k\right)-x_{j}^{*}\left(K\right)\right)}^{2}$$

where, $x_{j}$ shows the actual value, $x_{j}^{*}$ defines the acceptable values, and m shows the stages' number in the dataset training. The primary objective of this research is to make a strong optimized NN (ANN/IRFO) model as a device for the prediction of energy demand transportation.

#### 2.3.2 Application in transportation estimation demand

Today, energy plays a special role in improving the quality of life, development, and economic well-being of societies. Optimal use and proper policy-making increase the ability of managers in the energy need of the transport section. Because any planning in this area requires knowledge of the current consumption situation and its future trends. The need to predict the future trend has led to the application of different methods with the aim of more accurate prediction. Awareness of the better forecasting model is very important because of the impact it has on implementing policies and how successful they are. Considering the importance of needed energy in the transport section, in this research, by combining artificial neural networks with the IRFO algorithm an accurate method for predicting wanted energy in the section of transportation system could be introduced. ANN model implements randomly. The most appropriate solution to obtain satisfactory results for needed energy prediction in the transport section is the application of optimization algorithms. The main advantage of meta-algorithms is the assurance of results and the elimination of irrelevant, unnecessary, and inaccurate information. Also, the IRFO algorithms reduce computational complexity and enhance the ANN's effectiveness for forecasting the needed energy. The IRFO improves the error value in the prediction. It minimizes the error value and provides the desired result. The IRFO by optimizing the value of socio-economic parameters involved in simulating transportation electricity demand can increase forecast accuracy. Fig. (3) Shows a diagram of energy demand prediction in the transportation sector by the ANN\IRFO process.

**Fig. 3:** Diagram of energy demand prediction in the transportation sector by ANN\IRFO process.

### 2.4 The case study

China is a country of about 1.4 billion people located in the East Asian region, making it the most populous country on the globe. China is located at 39°55′ N, 116°23′ E. China does cover around $3.7\times 10^{6}$ square miles. It is also the third-biggest economy with regard to GDP. China's growing population and the advancement of industry and economic development have led to an increasing need for vehicles, especially in recent decades. China has the most motor vehicles in the world.

### 2.5 Data collection

Accurate forecasting of transportation estimation energy demand does depend on the precise assessment of ANN/IRFO technique variables. The results of processing the parameters foretell energy need in the transport section, which is the output variable in ANN/IRFO model. Transportation energy demand modeling parameters include population, GDP, and the vehicles’ number. The reason for using these three parameters is the most impact of these parameters in predicting the energy need in the transport section.

GDP, population, and the number of vehicles on the road all have complex relationships. The increase in vehicle numbers is often correlated with both population growth and GDP growth. Urbanization, government policies, and the transportation system are some of the other factors. Population growth often leads to increased energy demand in the transportation sector, both for individual trips and for the movement of commodities. As a result of this demand, the number of vehicles on the road may increase. Furthermore, an expanding economy, which is calculated by GDP, often results in increased individual income and increased demand for products and services, both of which contribute to an increase in the number of vehicles on the road. To effectively forecast transportation energy demand, a thorough understanding of the relationship between GDP, population, and vehicle numbers is required. These features, as explained below, can help estimate energy consumption in the transportation industry.

Population: Forecasting the population size of a country is very important in determining its energy demands. Population growth usually leads to the transportation of more products and people, which in turn increases energy demand. As a result, as the population increases, transportation energy demand will also increase.

GDP: A country's economic output is measured by its Gross Domestic Product (GDP). It contains every product and service created in a nation over a specific time frame. A greater GDP often translates into increased economic activity, which includes more transportation of both people and products, increasing energy demand. As a result, transportation energy demand is predicted to rise along with GDP.

Number of vehicles: Another important variable in predicting energy demand is the number of vehicles on the road. The number of vehicles on the road increases fuel consumption, which increases the demand for energy. As a result, the energy demand of the transportation sector is expected to increase along with the number of vehicles. The demand for vehicles is closely related to the demand for transportation energy. This necessity is caused by population increase, urbanization and economic growth. The increase in population causes more people to migrate to cities and thus increase the demand for transportation energy.

GDP data are collected from the Organization of Economic Co-operation and Development (OECD) [51]. The population data from the Statistical Institute of China [52]. The information on the vehicles’ number [53]. The energy need claims from the last 20 years are also collected from the 2020 report of China Electrical Energy Transmission Company [54]. The information about the input parameters is shown in Appendix I.

## 3 The discussion and result

### 3.1 Suggested algorithm validation

The IRFO performance validation has been illustrated in Table 3. This validation utilized the Average and Standard Deviation (SD) values to prove the performance of the proposed method.

**Table 3:** The validation results of the suggested model.

Test function	Metric	GA [48]	MVO [49]	SHO [42]	RFO [43]	IRFO
$F_{1}$	Average	7.13 E−10	6.04 E−13	4.98 E−15	3.19 E−18	1.46 E−19
	SD	7.31E-11	5.29E-14	4.81E-16	3.06E-19	2.05E-20
$F_{2}$	Average	38.32	11.93	7.97	3.16	0.0001
	SD	31.11	11.85	9.12	6.83	0.0001
$F_{3}$	Average	1.94	1.83	0.93	0.43	0.031
	SD	1.45	1.34	1.19	0.094	0.054
$F_{4}$	Average	3.36E-5	2.025	1.121	1.047	1.002
	SD	0.045	0.01	0.009	0.006	0.004
$F_{5}$	Average	0.51	0.51	0.51	0.51	0.51
	SD	1.33E-9	4.31E-10	3.12E-11	5.28E-12	7.05E-14

According to the results in Table 3, the IRFO has the lowest value for the objective functions compared to other optimization processes. The IRFO optimizer has a minimal SD, indicating that the outputs generated after 20 runs have highly accurate and reliable. As a result, the IRFO optimizer can provide a suitable and robust technique to forecast transportation energy demand. Therefore, the IRFO optimizer can provide verified and accurate results by achieving the lowest SD value. As a result, decision-makers and managers can employ the IRFO optimizer's prediction to make informed decisions about energy management and sustainability in the transportation industry. According to the data obtained, it can be indicated that the IRFO approach offers the following advantage compared with other methods.

1) The IRFO optimizer is the most accurate due to the lowest variance, which makes convergence more efficient in the optimal solution for forecasting energy demand in the transportation sector.
2) The IRFO optimizer outperformed other optimization techniques due to its reliability, precision, and stability. It is the best-suited strategy for estimating energy consumption in the transportation industry due to these benefits.

As a result, decision-makers and managers can depend on IRFO Optimizer to provide precise and reliable energy demand estimates. The suggested model allows them to make informed decisions regarding energy management and sustainability in the transportation industry. Generally, the study's findings emphasize the need of selecting a reliable and precise optimization algorithm for energy demand prediction in the transport industry, with the IRFO optimizer highlighted as a particularly useful tool for this purpose.

### 3.2 Simulation socio-economic using ANN/IRFO

The social and economic parameters and the number of vehicles are estimated by different models for the years 2006–2020. Fig. 4, Fig. 5, Fig. 6 shows the estimation results of indicators by different models. Also, the RMSE error rate of studied models has been calculated in comparison with the actual value. The RMSE error value of models has been shown in Fig. (7).

**Fig. 4:** The GDP value simulation.

**Fig. 5:** The population value simulation.

**Fig. 6:** The vehicle-number value simulation.

**Fig. 7:** The RMSE value of parameters.

The simulation results for each parameter for the current period demonstrated that, among the utilized models, the offered model of this research has the best simulation. The intention for this accuracy enhancement and reduction of errors in simulating socio-economic parameters is to solve optimization problems by using the IRFO optimization algorithm. Because by solving problems like being stuck in the optimal local area and the early convergent situation of the optimization, the efficiency of the model to simulate the desired goal increases. In addition, the RMSE error value of the parameters showed that, among the parameters, the number of vehicles and populations had the lowest RMSE error value compared to other parameters. Therefore, the most effective parameter in the energy demand prediction of the transpiration sector belongs to the number of vehicles. According to the exact simulation of the parameters by the proposed model, it can be concluded that this model has the most ability to simulate actual current energy demand and predict future energy needs. Fig. (8) does show the simulation of energy demand by diverse models. The results show that the model IRFO has the closest amount to the real one, so the IRFO approach is used to predict parameters and future energy demand.

**Fig. 8:** Simulation energy demand transportation by studied approach.

The suggested technique has been used to predict the growth rate of each of the parameters for the forthcoming 20 years in the following sector. Fig. (9) shows forecasting the growth of parameters affecting energy demand transportation for the next 20 years.

**Fig. 9:** Prediction of the growth of parameters.

The observations showed that the GDP, population, and vehicle quantity increased on average by 3.3 %, 2.4 %, and 2.1 %, respectively. The GDP, population, and vehicle numbers predicted by the model IRFO for the next 20 years have been predicted by 5.5 %, 4.8 %, and 4.2 %, respectively. Based on the results obtained from these parameters, it can be concluded that energy demand for transportation based on the three effective factors of GDP, population, and vehicle quantity can have an increasing trend. Fig. (10) shows the energy demand forecast for 2041.

**Fig. 10:** Energy demand prediction.

The results of forecasting energy demand transportation using the model IRFO showed that by 2041, the trend of energy demand transportation will be on the increase because of the growth in population, GDP, and the number of vehicles. With increasing GDP, the level of welfare and expectations of society will increase, and as the population grows, so will the demand for vehicles, which in turn will increase the need for energy to supply vehicles. Therefore, managers should be able to meet the need for energy by considering appropriate programs.

The achievement of The techniques utilized in the paper gives an effective strategy for forecasting energy demand in China's transportation industry. In estimating energy demand, the ANN model is better than other models when optimized with the Improved Red Fox Optimizer (IRFO). The LF technique and circular mapping-based chaotic process in the IRFO assist to avoid various optimization limitations, such as being trapped in the local optimum region.

Considering the enhancement of data quality, which leads to an augmented precision of forecasts, it is recommended to use a more extensive range of data in forthcoming research endeavors relative to the ongoing study to scrutinize energy demand. Furthermore, to elevate the accuracy of prognostications, a merged approach of classical and metaheuristic optimization can be employed. Even though classical estimation methods are more intricate and time-consuming, they are capable of producing absolute optimal outcomes, whereas metaheuristic methods can solve the most complex optimization difficulties in the shortest duration, but with an approximation of optimal results. Consequently, the combination of classical and metaheuristic methods can be utilized in the future to predict energy demand. This amalgamation would result in the achievement of highly accurate predictions and lead to a general advancement in the field of energy forecasting. Nonetheless, this approach would require further examination.

## 4 Conclusion

The primary objective of this study was to forecast the energy demand in the transportation sector of China for the next two decades. Given the crucial importance of accurately predicting energy demand in this sector, an optimized Artificial Neural Network (ANN) model was utilized. The Improved Red Fox Optimizer (IRFO) was used to optimize the ANN model. The proposed technique tackles some optimization drawbacks, such as being trapped in the local optimal region, by providing the LF method (Lévy flight) and a circular mapping-based chaos mechanism. The results of the estimates of energy demand for transportation by different models showed that the IRFO performed significantly better than the other models. Also, the results predicted by the ANN/IRFO model showed that the effective parameters for predicting energy demand have an increasing trend. The population, Gross Domestic Product (GDP), and number of vehicles have increased by almost 5.5 %, 4.8 %, and 4.2 %, respectively. Also, the trend of energy demand in transportation was increasing due to the increase of three effective parameters.

## Funding

This work was supported by Sichuan Province Luzhou city of Stars science and technology planning project (2021-JYJ-97), and scientific research and innovation team construction project of Luzhou vocational and Technical College (2021YJTD07).

## Data availability statement

No data was used for the research described in the article.

## CRediT authorship contribution statement

**Yijie Liu:** Formal analysis, Resources, Software, Writing – review & editing. **Gongxing Yan:** Conceptualization, Methodology, Software, Writing – review & editing. **Andrea Settanni:** Conceptualization, Data curation, Formal analysis, Resources, Software, Writing – original draft, Writing – review & editing.

## Declaration of competing interest

The authors declare that they have no known competing financial interests or personal relationships that could have appeared to influence the work reported in this paper.

## Figures and Tables

**Table 1:** Data needed to forecast energy need and transportation

Years	Energy demand (TWh)	GDP (Billions U.S. dollars)	Population (Billions of people)	Vehicle-number (Million)
2006	19.51	2754.11	1.311	51
2007	19.83	3555.7	1.318	64
2008	20.01	4577.4	1.325	73
2009	20.38	5088.99	1.331	85
2010	20.62	6033.99	1.338	90.86
2011	20.93	7492.26	1.344	104.5
2012	21.94	8539.47	1.351	120
2013	22.32	9625.04	1.357	137
2014	23.18	10524.21	1.364	154
2015	24.91	11113.53	1.371	172
2016	25.33	11228.08	1.379	194
2017	25.97	12265.32	1.386	217
2018	26.65	13841.9	1.393	240
2019	28.34	14,340.9	1.398	258
2020	30.15	14722.84	1.439	281
